RETRACTED

# circZC3HAV1 Regulates TBC1D9 to Affect the Biological Behavior of Colorectal Cancer Cells

**DOI:** 10.1155/2022/7386946

**Published:** 2022-09-16

**Authors:** Jianxian Zhang, Yan Xue, Hengling Gao, Yunxi Yu, Huabin Cheng, Xukun Lv, Ke Ke

**Affiliations:** ^1^Department of Gastrointestinal Surgery, The Second People's Hospital of Liaocheng, Liaocheng, 252600 Shandong, China; ^2^Department of Gastroenterology, The Second People's Hospital of Liaocheng, Liaocheng, 252600 Shandong, China; ^3^Department of Emergency, Huangshi Hospital of Traditional Chinese Medicine (Municipal Infectious Disease Hospital), Huangshi, China; ^4^Puai Hospital of Huangshi Central Hospital of East Hubei Medical Group, Affiliated Hospital of Hubei Institute of Technology, Huangshi, 435000 Hubei, China

## Abstract

**Background:**

Colorectal cancer (CRC) is one of the most frequently diagnosed cancers all over the world, which accounts for a large proportion of cancer-associated deaths. The regulatory function of circular RNAs (circRNAs) has been affirmed in diverse cancers. circ_0082628, named circRNA zinc finger CCCH-type containing antiviral 1 (circZC3HAV1), has been discovered to be significantly downregulated in CRC tissues. Nevertheless, the function and mechanism of circZC3HAV1 in CRC remain unclear.

**Purpose:**

We targeted at studying the specific role and mechanism of circZC3HAV1 in CRC cells.

**Methods:**

The expression of the genes was detected by quantitative real-time polymerase chain reaction (qPCR). The binding relationship among different genes was verified by mechanism assays. Functional assays were carried out to reveal the role of different RNAs in CRC cell malignant behaviors.

**Results:**

circZC3HAV1 was significantly downregulated in CRC cells. circZC3HAV1 overexpression hampered CRC cell migratory and invasive abilities. As for the mechanism, circZC3HAV1 competitively bound with microRNA-146b-3p (miR-146b-3p) to enhance the expression of TBC1 domain family member 9 (TBC1D9). Rescue assays demonstrated circZC3HAV1 sponged miR-146b-3p and upregulated TBC1D9 to restrict migration and invasion of CRC cells.

**Conclusion:**

circZC3HAV1 could upregulate TBC1D9 via absorbing miR-146b-3p, consequently inhibiting migratory and invasive capabilities of CRC cells.

## 1. Introduction

Colorectal cancer (CRC) is a common diagnosed malignancy in both genders in the world. Although improvements have been achieved in diagnostic and therapeutic methods, CRC still leads to cancer-related deaths significantly [1]. Hence, it is important to understand the potential regulatory mechanism underlying CRC in order to develop effective treatments.

Circular RNAs (circRNAs) belong to noncoding RNAs with a covalently closed structure that are derived from back-splicing [2]. The regulatory function of circRNAs has been affirmed in diverse cancers. For instance, circRNA_0000392 contributes to CRC development through the miR-193a-5p/PIK3R3/AKT axis [3]. Exosomal circPACRGL promotes CRC progression through the miR-142-3p/miR-506-3p/TGF-*β*1 pathway [4]. Moreover, circHIPK3 prompts CRC growth and metastasis via sponging miR-7 [5]. Therefore, to find out a novel circRNA and uncover its role and potential regulatory mechanism in CRC are of interest.

RETRACTED

MicroRNAs (miRNAs) refer to small noncoding RNAs which could repress or degrade target messenger RNAs (mRNAs) [6]. mRNAs have become a promising class of drugs for all kinds of therapeutic applications in the past few years [7]. It has been reported that the competing endogenous RNA (ceRNA) network (circRNA-miRNA-mRNA) is implicated in various cancers including squamous cell carcinoma [8], melanoma [9], and lung adenocarcinoma [10]. CRC has been reported to be regulated by ceRNA pattern as well. For example, circ_001680 influences the proliferative and migratory abilities of CRC through regulating BMI1 mRNA targeted by miR-340 [11]. circCAMSAP1 facilitates CRC tumor growth via modulation of the miR-328-5p/E2F1 pathway [12]. Furthermore, hsa_circRNA_002144 sponges miR-615-5p to upregulate LARP1, consequently promoting CRC progression [13]. Hence, whether ceRNA network is involved in the malignant behaviors of CRC cells is worthy to be unveiled.

In summary, the main focusing point of our research was to study the role and underlying mechanism of a novel circRNA in CRC, which might provide new potential biomarkers or therapeutic targets for CRC.

## 2. Materials and Methods

### 2.1. Cell Culture

Human CRC cell lines (NCI-H508, RKO, and CW-2) were procured from Cell Resource Center, Peking Union Medical College. Human colonic epithelial cell line FHC was procured from Kunming Cell Bank, Chinese Academy of Sciences. 293T cells were acquired from National Institutes for Food and Drug Control. NCI-H508 and CW-2 cells were cultivated in RPMI 1640 (w/o Hepes)+10% fetal bovine serum (FBS). RKO cells were cultured in Minimal Essential Medium-Earle's Balanced Salt Solution (MEM-EBSS) +10% FBS. FHC cells were left to grow in basic medium+10% FBS. And 293T cells were cultivated in RPMI-1640 medium+10% FBS. All the cells were cultured with 5% CO_2_ at 37°C.

### 2.2. Plasmid Transfection

In order to overexpress circZC3HAV1, pcDNA3.1-circZC3HAV1 vectors were synthesized in advance. Empty pcDNA3.1 worked as the negative control (NC), while for the overexpression of miR-146b-3p, miR-146b-3p mimics was used. For the knockdown of lemur tyrosine kinase 2 (LMTK2), TBC1 domain family member 9 (TBC1D9), tumor protein p53 inducible nuclear protein 2 (TP53INP2), and specific short hairpin RNAs (si-RNAs) were devised and constructed with nontargeting si-RNA (si-NC) as control. In accordance with the protocols, the transfections were performed with Lipofectamine 2000 (Invitrogen).

RETRACTED

### 2.3. Quantitative Real-Time Polymerase Chain Reaction (qPCR)

QPCR analysis was conducted based on previous protocol [14]. Based on the guidance of TRIzol reagent (Takara, Japan), the extraction of total RNA from cells was completed. The complementary DNA (cDNA) for miRNAs was generated utilizing TaqMan™ MicroRNA Reverse Transcription Kit, while the cDNA for circRNAs and mRNAs was obtained by means of PrimeScript RT Reagent Kit. QPCR reaction was conducted with SYBR Green PCR Kit followed by 2^-*ΔΔ*Ct^ method. *β*-Actin or U6 was used as internal reference for miRNA or circRNA/mRNA.

### 2.4. Transwell Assay

Transwell assay was conducted as previously described [15]. To assess the migratory ability, CRC cells were fixed on the upper part of 24-well Transwell chambers without Matrigel. As for invasion assay, the top compartment was coated with Matrigel. The lower chambers were added with FBS. After 24 h, cells that successfully migrated or invaded into the lower compartment were fixed by methanol for 15 min. In the end, cells stained by crystal violet was subjected to microscope observation.

### 2.5. Cell Counting Kit-8 (CCK-8) Assay

Cell viability was assessed via CCK-8 analysis following previous research [14]. CW-2 and RKO cells were seeded to 96-well plates for cultivation. Next, 10 *μ*l of CCK-8 solution (Dojindo, Kumamoto, Japan) was added for 1 h incubation. Absorbance at 450 nm was detected with the microplate reader.

### 2.6. Wound Healing Assay

The assay was performed as previously described [16]. CW-2 or RKO cells were plated in 24-well plates. After cell confluence reached over 80%, pipette tip was taken to scratch the surface of cell layer. Afterwards, phosphate-buffered saline (PBS) was utilized to wash the detached cells. Subsequently, the width of wound at 0 h was captured and recorded. Next, cells were cultured for another 24 h, and the wound width was photographed and recorded.

### 2.7. Flow Cytometry Analysis

This assay was conducted following precious description [16]. Transfected CRC cells were harvested and rinsed with PBS. Later, cells were double stained with Annexin V-FITC/PI Apoptosis kit. Apoptotic rate of the cells was evaluated by a Cytoflex flow cytometer, and the data collected were analyzed with FlowJo software.

### 2.8. Fluorescence In Situ Hybridization (FISH) Assay

FISH assay was carried out according to published research [17]. The FISH probe prepared for circZC3HAV1 localization was synthesized by Ribobio (Guangzhou, China). The sequence of specific FISH probe was biotin-TTAATTACTTGATAAAGAAT-biotin. FISH probes were incubated with CW-2 and RKO cells in hybridization buffer. Afterwards, nuclei were counterstained with 4′,6-diamidino-2-phenylindole (DAPI). Finally, confocal laser scanning microscope (Zeiss LSM7 DUO) was adopted to observe the subcellular localization of circZC3HAV1.

RETRACTED

### 2.9. Subcellular Fractionation Assay

PARIS™ Kit was applied to carry out the experiment in CW-2 and RKO cells. After centrifugation, cells were treated with cell disruption buffer. Eventually, the level of circZC3HAV1 in the cytoplasm and nucleus was examined by qPCR. *β*-Actin or U6 was used as nuclear or cytoplasmic control.

### 2.10. RNA Pull Down Assay

The Pierce™ RNA 3′ End Desthiobiotinylation Kit was used for conducting the experiments. miR-146b-3p with wild-type (WT) or mutant (MUT) sequence was marked with biotin. Cell lysates of 1 × 10^6^ cells were incubated with bio-NC, bio-miR-146b-3p-WT, or bio-miR-146b-3p-MUT for 1 h. Afterwards, precipitated RNAs were purified. The enrichment of circZC3HAV1 was examined by qPCR.

### 2.11. RNA Binding Protein Immunoprecipitation (RIP)

This assay was performed as previously described [18]. Using Magna RIP RNA-Binding Protein Immunoprecipitation Kit, RIP assay was carried out. CW-2 and RKO cells were lysed by RIP buffer first and then cocultured with anti-argonaute-2 (AGO2) or anti-immunoglobulin G (IgG) (NC group). Next, magnetic beads were added into cell lysates for incubation at 4°C, followed by RNA expression analysis through qPCR.

### 2.12. Luciferase Reporter Assay

The assay was carried out as previously described [18]. Full-length of TBC1D9 3′ untranslated regions (3′UTR) covering wild-type or mutant miR-146b-3p binding sites was inserted into pmirGLO luciferase vectors to construct pmirGLO+TBC1D9 3′UTR-WT/MUT. Similarly, pmirGLO+circZC3HAV1-WT/MUT plasmids were obtained. miR-146b-3p mimics or NC mimics was cotransfected with the abovementioned plasmids into CRC cells. After 48 h transfection, the luciferase activity was analyzed, utilizing the dual-luciferase reporter assay system.

### 2.13. Statistical Analyses

Each experiment was conducted in triplicate. Experimental data were subject to SPSS software analysis and shown as mean ± standard deviation (SD). The differences between two groups were compared by Student's *t*-test, while the differences among multiple groups were assessed by one-way or two-way analysis of variance (ANOVA). Statistic difference with *P* value less than 0.05 was regarded to be statistically significant.

RETRACTED

## 3. Results

### 3.1. circZC3HAV1 Is Significantly Downregulated in CRC Cells

At first, we used the GEO database to look for the circRNAs that were remarkably downregulated in CRC tissues in comparison with normal tissues. Under the conditions of *P* < 0.05 and |logFC| ≥ 2, 8 circRNAs were picked. Among the 8 circRNAs, hsa_circ_0009361 and hsa_circ_0003266 have been studied in CRC [19] [20]; hsa_circ_0005927 has been studied in gastric cancer [21]; hsa_circ_0043278 has been studied in lung cancer [22]; and hsa_circ_0000775 has been studied in Alzheimer disease [23]. Therefore, hsa_circ_0012634, hsa_circ_0082628, and hsa_circ_0020934 were chosen as candidates. The bioinformatics prediction of the candidate circRNA expression in CRC tissues and normal tissues was displayed (Figure 1(a) and Figure S1A–C). Then, the expression of the three circRNAs in human normal colorectal epithelial cells (FHC) and CRC cell lines (CW-2, RKO, and NCI-H508) was measured by qPCR. The result elucidated that the expression level of circ_0082628 was obviously lower in CRC cell lines than that of the other two circRNAs (Figure 1(b)). Therefore, circ_0082628 was chosen for further experiments. As its host gene is ZC3HAV1, we named it as circZC3HAV1 in our study. Loop formation diagram of circ_0082628 was shown in Figure 1(c). After CW-2 and RKO cells were treated with Actinomycin D (ActD), the expression of circZC3HAV1 and ZC3HAV1 mRNA was examined by qPCR. The outcome uncovered that the expression of ZC3HAV1 mRNA was noticeably decreased, while that of circZC3HAV1 was hardly changed (Figure 1(d)). Moreover, the expression of circZC3HAV1 and *β*-actin was examined by qPCR in CW-2 and RKO cells with RNase R treatment. We found that the circZC3HAV1 expression had no significant change, while *β*-actin expression dramatically declined (Figure 1(e)). To summarize, circZC3HAV1 has a stable loop structure and displays a significantly lower expression in CRC cells.

### 3.2. circZC3HAV1 Overexpression Impedes CRC Cell Migration and Invasion

In this part, we mainly delved into the specific influence of circZC3HAV1 on CRC cell malignant behaviors. At first, the high overexpression efficiency of pcDNA3.1-circZC3HAV1 was validated by qPCR in CRC cells (Figure 2(a)). Next, wound healing assay was done to reveal the migratory condition of CRC cells when circZC3HAV1 was overexpressed. We found that circZC3HAV1 overexpression inhibited cell migration (Figure 2(b)). Transwell assays were then implemented for the assessment of cell migratory and invasive abilities. The experimental results showed that overexpressing circZC3HAV1 restricted cell migration and invasion (Figures 2(c) and 2(d)). Moreover, qPCR was utilized to test the expression of invasion-linked factors (MMP2 and MMP9). We noticed expression of these factors decreased upon circZC3HAV1 augment (Figure 2(e)). CCK-8 was utilized to uncover the influence of overexpressing circZC3HAV1 on CRC cell proliferation. We found that circZC3HAV1 up-regulation had no obvious influence on cell proliferation (Figure S1D–E). Finally, flow cytometry analysis was taken to measure the apoptosis rate of the cells after overexpressing circZC3HAV1. The outcomes elucidated that there was no obvious change in cell apoptosis (Figure S1F). To conclude, circZC3HAV1 overexpression hinders migration and invasion of CRC cells.

RETRACTED

### 3.3. circZC3HAV1 Sponges miR-146b-3p in CRC Cells

As revealed in Figure 2, circZC3HAV1 augment inhibited CRC cell invasive and migratory abilities *in vitro*. Hence, we tried to uncover the downstream regulatory mechanism of circZC3HAV1 in CRC cells. Based on the results of subcellular fractionation and FISH assays, circZC3HAV1 was mainly distributed in cytoplasm (Figures 3(a) and 3(b)). Then, RIP assay showed circZC3HAV1 was enriched in anti-AGO2 in both CW-2 and RKO cells (Figure 3(c)), indicating circZC3HAV1 might regulate the downstream genes through ceRNA pattern. circBank database (http://www.circbank.cn/) was used to predict the miRNAs which might bind to circZC3HAV1. The top 10 miRNAs (in a descending order of binding site number) were selected (Figure 3(d)). Among these miRNAs, miR-1200, miR-5587-5p, miR-6828-5p, miR-1914-5p, and miR-302b-3p have not been studied in cancers; miR-378a-5p, miR-1254, and miR-302a-3p have been proven to inhibit CRC progression [24–26]; miR-671-5p has been revealed to promote prostate cancer progression [27]; miR-146b-3p has been found to accelerate progression of liver cancer [28] and thyroid cancer [29]. Therefore, we chose miR-671-5p and miR-146b-3p as candidates. In CW-2 cells, the enrichment of the two miRNAs in Bio-circZC3HAV1 was detected after RNA pull down assay. The outcomes indicated that miR-146b-3p had the better binding ability with circZC3HAV1 (Figure 3(e)). Therefore, miR-146b-3p was chosen for the following experiments. Subsequently, we learned from the RIP result that circZC3HAV1 could bind to miR-146b-3p (Figure 3(f)). Moreover, RNA pull down assay outcome further proved the finding above that circZC3HAV1 could bind to miR-146b-3p (Figure 3(g)). In 293T cells, luciferase reporter assay was implemented to evaluate the circZC3HAV1 luciferase activity when miR-146b-3p was overexpressed. The data revealed that circZC3HAV1 could interact with miR-146b-3p as the luciferase activity declined upon miR-146b-3p augment (Figure 3(h)). Finally, the expression of miR-146b-3p was tested via qPCR before and after the overexpression of circZC3HAV1. It turned out the expression of miR-146b-3p had no obvious change (Figure 3(i)). To sum up, circZC3HAV1 competitively adsorbs miR-146b-3p in CRC cells.

RETRACTED

### 3.4. circZC3HAV1 Competitively Binds with miR-146b-3p to Restrain CRC Cell Migration and Invasion

The overexpression efficacy of miR-146b-3p mimics was tested by qPCR in CRC cells at first (Figure 4(a)). Then, in CW-2 and RKO cells with transfection of miR-146b-3p mimics, wound healing assay was done for assessing the cell migratory condition. It turned out miR-146b-3p overexpression promoted CRC cell migration (Figure 4(b)). The migratory and invasive abilities of CRC cells were analyzed by Transwell assays after overexpressing miR-146b-3p. The experimental outcomes proved that overexpressing miR-146b-3p could accelerate the migration and invasion of CRC cells (Figures 4(c) and 4(d)). After the upregulation of miR-146b-3p, qPCR was employed to test the expression of MMP2 and MMP9. The expression of the genes increased, which indicated that overexpressing miR-146b-3p accelerated CRC cell invasion (Figure 4(e)). Wound healing assay was implemented to monitor the CRC cell migration under diverse conditions. When circZC3HAV1 was overexpressed, the cell migration was inhibited, while the cotransfection of miR-146b-3p mimics offset its influence (Figure 4(f)). In addition, Transwell assays demonstrated the suppressive impact of circZC3HAV1 overexpression on cell migration and invasion was counteracted by miR-146b-3p augment (Figure 4(g)). The expression of MMP2 and MMP9 in CRC cells was detected by qPCR. The inhibited expression of MMP2 and MMP9 caused by pcDNA3.1-circZC3HAV1 was recovered by overexpressing miR-146b-3p (Figure 4(h)). In summary, circZC3HAV1 restricts CRC cell migration and invasion via competitively binds with miR-146b-3p.

### 3.5. circZC3HAV1 Regulates TBC1D9 Expression via Competitively Adsorbing miR-146b-3p

DIANA database (http://diana.imis.athena-innovation.gr/) was used to project the mRNAs that might bind to miR-146b-3p, and 15 mRNA candidates were projected (Figure 5(a)). Afterwards, we utilized UALCAN (http://ualcan.path.uab.edu/index.html) to search for the expression of 15 candidate mRNAs in colon adenocarcinoma (COAD) tissues and normal tissues (Figure S2A–O). As only LMTK2, TBC1D9, and TP53INP2 were significantly downregulated in COAD tissues, they were involved in the following research. The interference efficiency of candidate mRNAs was measured by qPCR in CRC cells. The results were shown in Figures 5(b)–5(d). After interfering LMTK2, the migration of CRC cells was detected through wound healing assays, and MMP2 and MMP9 expressions in CRC cells were detected by qPCR. Through the results above, we could conclude that LMTK2 interference had no significant influence on cell migration and invasion (Figures 5(e) and 5(f)). Next, the influence of TBC1D9 knockdown on the migration and invasion of CRC cells was detected via wound healing assays and qPCR. We found that interfering TBC1D9 could promote cell migration and invasion (Figures 5(g) and 5(h)). Moreover, results of wound healing and qPCR assays manifested TP53INP2 depletion had no obvious influence on cell migration and invasion (Figures 5(i) and 5(j)). Hence, we finally chose TBC1D9 as the target gene. In CRC cells, RIP assay result showed that circZC3HAV1, miR-146b-3p, and TBC1D9 were all enriched in anti-AGO2 (Figure 5(k)). Luciferase reporter assay was done to measure the luciferase activity in 293T cells. We found after transfection of miR-146b-3p mimics, the luciferase activity of TBC1D9 3′UTR was decreased, while cotransfection of pcDNA3.1-circZC3HAV1 totally recovered the luciferase activity (Figure 5(l)). In CW-2 cells, wound healing assay was carried out to detect the CRC cell migration. We noticed suppressed cell migration caused by circZC3HAV1 overexpression was reversed totally by inhibiting TBC1D9 (Figure 5(m)). Transwell assay was conducted to detect CRC cell migratory and invasive capabilities. When circZC3HAV1 was overexpressed, CRC cell migratory and invasive abilities were inhibited, while TBC1D9 inhibition could totally abrogate the suppressive impact (Figure 5(n)). Furthermore, based on qPCR analysis, decreased MMP2 and MMP9 expression caused by pcDNA3.1-circZC3HAV1 was restored by inhibiting TBC1D9 (Figure 5(o)). Taken together, circZC3HAV1 sponges miR-146b-3p to upregulate TBC1D9, thus impeding CRC cell migration and invasion.

RETRACTED

## 4. Discussion

CRC is the third commonest cancer globally and causes cancer-linked death in both genders [30]. There exist multiple conventional treatment options for CRC ranging from simple endoscopic polypectomy, radio-chemotherapy, to complex chemotherapeutical regimen combined with drugs, but these treatments all have some disadvantages and side effects [31] [1]. During the past years, the management of CRC has been advanced. However, metastatic CRC is still difficult to treat. A deeper understanding of the pathways involved in the malignant processes of cancer cells has driven the development of targeted therapies [32]. Therefore, it is in an urgent need to explore more potential targets for CRC to improve its treatment.

circRNAs are noncoding RNA family members that have a close structure. The function of circRNAs has been affirmed in diverse diseases [33]. In the recent five years, the studies on the features and roles of circRNAs in CRC are on the rise. For instance, circRNA_0000392 accelerates CRC progression via miR-193a-5p/PIK3R3/AKT axis [3]. Moreover, it has been validated that circDDX17 functions as a tumor suppressor in CRC [34]. As a newly found circRNA, circZC3HAV1 was found to be evidently downregulated in CRC cells, and circZC3HAV1 overexpression inhibited CRC cell migration and invasion.

circRNAs can act as ceRNAs to indirectly modulate gene expression via shared miRNAs [35]. The existence of circRNA-associated ceRNA network (circRNA-miRNA-mRNA) has been identified in various cancers, including CRC. For example, circ3823 has been uncovered to act as a ceRNA of miR-30c-5p to restrain the inhibiting impact of miR-30c-5p on its target TCF7 mRNA, which eventually promotes CRC progression [36]. In the present research, we first found that circZC3HAV1 could bind to miR-146b-3p in a ceRNA manner. As reported, elevated expression of miR-146b-3p in CRC tissues and cells is linked to unfavorable overall survival [37]. Consistent with this literature, our study confirmed miR-146b-3p overexpression facilitated CRC cell migratory and invasive processes. Subsequently, we discovered that TBC1D9 was the downstream mRNA of miR-146b-3p. After a series of mechanism and rescue assays, it was unveiled that circZC3HAV1 could restrict the malignant behaviors of CRC cells via regulating the miR-146b-3p-TBC1D9 pathway.

Due to the limited time and experimental materials, *in vivo* assays and clinical samples are not involved in this research. However, there are still some innovative points in our study. Our study is the first to verify that circZC3HAV1 plays an oncogenic part in CRC cells. Moreover, the finding that circZC3HAV1 influences invasion and migration of CRC cells through regulating the miR-146b-3p/TBC1D9 axis is also new. We hope our study might provide useful information for relevant research on CRC.

## Figures and Tables

**Figure 1:** circZC3HAV1 has low expression level and a stable loop structure in CRC cells. (a) Three candidate circRNAs were picked from the GSE142837 dataset under specific conditions and showed in a volcano plot. (b) QPCR detected the expression of candidate circRNAs in human normal colorectal epithelial cells FHC and CRC cells (CW-2, RKO, and NCI-H508). (c) The diagram of hsa_circ_0082628 formation (ZC3HAV1 as the host gene) was demonstrated. (d) circZC3HAV1 and ZC3HAV1 expression levels were measured by qPCR in CRC cells treated with ActD. (e) circZC3HAV1 expression was measured by qPCR in CRC cells treated with RNase R. ^∗^*P* < 0.05; ^∗∗^*P* < 0.01.

RETRACTED

**Figure 2:** circZC3HAV1 upregulation contributes to the inhibition of CRC cell migration and invasion. (a) The overexpressing efficiency of pcDNA3.1-circZC3HAV1 was detected by qPCR. (b) Wound healing assay evaluated the effect of circZC3HAV1 on CRC cell migration. Scale bar: 100 *μ*m. (c, d) Transwell assay was conducted to measure the migratory and invasive abilities of CRC cells upon circZC3HAV1 upregulation. Scale bar: 100 *μ*m. (e) QPCR was implemented to examine the expression of MMP2 and MMP9 in CW-2 and RKO cells upon circZC3HAV1 overexpression. ^∗∗^*P* < 0.01.

**Figure 3:** circZC3HAV1 competitively binds to miR-146b-3p in CRC cells. (a,b) The localization of circZC3HAV1 in CRC cells was detected through subcellular fractionation and FISH assays. Scale bar: 10 *μ*m. (c) RIP assay was conducted to detect the enrichment of circZC3HAV1 in anti-AGO2. (d) circBank database was used to project the potential miRNAs which might bind to circZC3HAV1. (e) The binding affinities between circZC3HAV1 and candidate miRNAs were evaluated by RNA pull down assay. (f) RIP assay was performed to detect the enrichment of circZC3HAV1 and miR-146b-3p in anti-AGO2 by RIP assay. (g) The binding of circZC3HAV1 and miR-146b-3p was tested by RNA pull down assay. (h) In 293T cells, luciferase reporter assay was implemented to examine the luciferase activity of circZC3HAV1 when miR-146b-3p was upregulated. (i) The miR-146b-3p expression was examined by qPCR before and after the overexpression of circZC3HAV1 in CRC cells. ^∗∗^*P* < 0.01.

**Figure 4:** circZC3HAV1 regulates CRC cell migration and invasion by sponging miR-146b-3p. (a) The overexpression efficacy of miR-146b-3p mimics was measured by qPCR in CRC cells. (b) Wound healing assay was utilized for detecting the migratory capability of CRC cells in response to miR-146b-3p mimics. Scale bar: 100 *μ*m. (c, d) The migratory and invasive abilities of CRC cells were detected by Ttranswell assays after overexpressing miR-146b-3p. Scale bar: 100 *μ*m. (e) After the overexpression of miR-146b-3p, qPCR was utilized to detect the expression of MMP2 and MMP9. (f) Wound healing assay was performed to detect CRC cell migration under different conditions. (g) Migratory and invasive processes of CRC cells were evaluated by Transwell assays upon indicated conditions. (h) The expression of MMP2 and MMP9 in CRC cells transfected with different plasmids was detected by qPCR. ^∗∗^*P* < 0.01.

**Figure 5:** circZC3HAV1 regulates TBC1D9 expression via competitively adsorbing miR-146b-3p. (a) DIANA tools database was used to detect candidate mRNA that might bind to miR-146b-3p. (b, d) The interference efficiency of target mRNAs was measured by qPCR in CRC cells. (e) After LMTK2 downregulation, the migration of CRC cells was monitored in wound healing assays. Scale bar: 100 *μ*m. (f) After LMTK2 knockdown, MMP2 and MMP9 expressions in CRC cells were detected by qPCR. (g) After TBC1D9 deficiency, the migration of CRC cells was tested by wound healing assays. Scale bar: 100 *μ*m. (h) Upon TBC1D9 depletion, MMP2 and MMP9 expressions in CRC cells were detected by qPCR. (i) After downregulation of TP53INP2, the migration of CRC cells was examined via wound healing assays. Scale bar: 100 *μ*m. (j) After knockdown of TP53INP2, the expression of MMP2 and MMP9 in CRC cells was detected by qPCR. (k) The enrichment of circZC3HAV1, miR-146b-3p, and TBC1D9 were detected by RIP assay in CRC cells. (l) Luciferase reporter assay was carried out to detect the influence of circZC3HAV1 overexpression on the binding of TBC1D9 and miR-146b-3p in 293T cells. (m) CRC cell migration was detected by wound healing assay under different conditions. (n) Transwell assay was applied for assessing migration and invasion of CRC cells transfected with different plasmids. (o) MMP2 and MMP9 expressions were detected by qPCR in CW-2 cells transfected with indicated plasmids. ^∗∗^*P* < 0.01.

RETRACTED

## Data Availability

The data used to support the findings of this study are included within the article.

## Supplementary Materials

Supplementary 1 Figure S1. (A–C) The expression of candidate circRNAs was analyzed in adjacent normal and CRC tissues based on the GEO database (GSE142837). (D, E) CCK-8 assay was conducted to measure the influence of circZC3HAV1 augment on CRC cell proliferation. (F) Flow cytometry analysis was done to measure the apoptosis rate of CRC cells after overexpressing circZC3HAV1.

Supplementary 2 Figure S2. (A–O) UALCAN database was applied to project the expression of candidate target mRNAs in normal and CRC tissues.
